The article "Research on the Purification of Environmental Pollution by Biomaterials and Its Treatment Methods in the Development of Rural Cultural and Creative Industries" was retracted in 2023. Reasons: signs of a paper mill; suspected computer-generated content; unreliable results or conclusions; concerns about the data.

# Research on the Purification of Environmental Pollution by Biomaterials and Its Treatment Methods in the Development of Rural Cultural and Creative Industries

**DOI:** 10.1155/2022/1594081

**Published:** 2022-10-04

**Authors:** Ting Fan, Tianyou Fu, Qun Xu, Gazmir Gjoni

**Affiliations:** ^1^Institute of Human Geography, College of Tourism, Xi'an International Studies University, Xi'an, Shanxi, China; ^2^Shanghai Maritime University, Shanghai, China; ^3^Shandong University of Technology, Zibo, China; ^4^Autonomous University of Zacatecas, ZAC, Mexico

## Abstract

Since our country put forward the rural revitalization strategy, we have attached great importance to the construction and development of urban and rural areas. In recent years, we have continuously enhanced the driving force of development and further promoted rural reform. However, in the construction of rural cultural industry, how to purify environmental pollution is a key and difficult point. Through the comprehensive analysis of the role and effect of biomaterials in environmental pollution purification, this study compares the comprehensive role of different materials in environmental purification, compares the trend of environmental pollution in the development of rural industries in recent years, and analyzes the coupling degree of environmental pollution purification in different technological environments. Through the analysis, we can draw a conclusion that under the action of nanomaterials and biomaterials, some water pollution, air pollution, construction waste pollution, and noise pollution in industrial development have achieved good results and impact. Through continuous practice and research, it can be seen that biotechnology and materials can play a relatively good role in the environmental pollution control. And this treatment technology has the advantages of low cost, high efficiency, and no secondary pollution. It also plays an important role in the treatment of pollutants and the development of new energy. It conforms to the concept of sustainable development and environmental construction in the modern society and provides more reference data and research value for the future research and development prospects of nanomaterials and biomaterials in industrial development and environmental governance.

## 1. Introduction

With the rapid development of China's economy and society, rural revitalization and construction also follow the pace. No matter whether it is urban or rural, development is inseparable from industry, and the rural culture is the main force in the current creative industry. Based on cultural resources, develop creative industries. Wang et al. pointed out that rural cultural and creative industries are the use of people's traditional cultural resources. Under the concept of modern economic development, combined with the cultural and tourism industry model, rural cultural and economic activities and the development of rural culture should obtain new directions from culture, tourism, and science and technology [1]. Xie pointed out that while developing beautiful villages, we should improve traditional thinking and explore new industries in the development of cultural and creative industries. In this context, we should take cultural creativity and the tourism industry as the development direction to help rural cultural creativity, and the participation of the tourism industry helps to establish countermeasures for its sustainable development [2]. Zhang pointed out that with the continuous development of rural revitalization, new opportunities have been brought to the cultural and creative industry. The state has given strong support to rural economic and ecological construction, so it is very beneficial for the rural cultural and creative industry to build a brand [3]. Li et al. pointed out that under the revitalization and development of rural areas, the environmental pollution problems in rural areas have not been well treated, and the indiscriminate spraying of fertilizers and the residues of chemicals in agricultural production have caused serious pollution to the rural environment [4]. Peng et al. made a detailed analysis of sewage treatment technology according to green environmental protection organisms and ecology and pointed out that rural sewage treatment should focus on water purification [5]. Chao pointed out that nanomaterials have the advantage of a large specific surface area. In water treatment technology, the application of nano adsorption materials, nanomembranes, and catalysts is more efficient and safer in water treatment areas [6]. Zou et al. proposed that the application of biological nanocomposites can effectively adsorb, achieve photocatalysis, possess antibacterial mechanism, and remove heavy metals, organic dyes, drugs, inorganic salts, and other pollutants in water treatment, which can effectively solve the problem of traditional sewage treatment [7]. According to Sun et al., nanomaterial is not only a low-cost and ecological material but also can produce electron-hole pair separation and other properties under light, electricity, ultrasound, and other conditions. It has a good effect on wastewater treatment. Based on the characteristics of many pores and strong adsorption capacity, it can be reused [8]. Through the research on the purification of environmental pollution and treatment methods of biomaterials in the development of rural cultural and creative industries, this study points out that in the development of rural culture, environmental treatment is a necessary condition and the use of biomaterials to improve environmental pollution; it can more effectively improve the effect of rural environmental governance and promote the sustainable development of rural cultural and creative industries more efficiently.

## 2. Significance and Value of Rural Cultural and Creative Industries

Creative industry, also known as innovative economy, generally refers to the enterprises that have achieved development momentum in personal creativity and talent skills and use intellectual property rights to create more graduation opportunities and activities. With the rapid development of society, the development of rural cultural industry has not only made minor achievements in culture but also made breakthroughs in art. The development of cultural and creative industries is an important way to promote rural structural adjustment. The development of creative industries not only develops a new development space but also promotes employment and entrepreneurship, so that more people turn from consumers to operators or producers, resulting in a number of emerging industries, the construction of industrial chains, and the growth of the rural economy. This is new and increasingly occupies the total amount of the cultural industry, accelerating the cultural industry to become the most important channel for the development of China's future pillar industry. The development of culture through industrialization and the use of cultural elements to promote the economy has not only improved the national economy but also made greater contributions to the dissemination and protection of our culture, thereby enhancing the creativity of culture.

## 3. Environmental Pollution in the Development of Rural Cultural and Creative Industries

With the development of rural revitalization and the continuous promotion of rural ecological construction, the increasingly serious pollution of rural environment and water resources has been widely concerned by the society. In the development of rural culture and creativity, rural areas have brought benefits, while environmental problems have also been affected. The garbage discarded casually has brought a great burden, which is full of peculiar smell around, and the white garbage of kitchen garbage, once burned, is also very serious to air pollution. It not only affects physical and mental health but also affects beauty. In addition, the cultural industrial park has a large flow of people, and the domestic wastewater industry also causes varying degrees of pollution to rural rivers.

Figure 1 shows that many environmental pollution problems caused by the development of rural creative industries in China are becoming more and more serious. With the construction of modern concepts and equipment and facilities, more environmental pollution is formed in the construction materials, construction equipment, construction noise, and other aspects. In this case of large environmental pollution, it has brought greater damage to rural residents and the ecological environment. It is not conducive to economic construction and residents' life. Solving the problem of rural environmental pollution purification is the primary problem and difficulty.

## 4. Treatment Methods of Environmental Pollution in Rural Cultural and Creative Industries

### 4.1. The Role of Biological Materials in Purifying Pollution

With the continuous development of biotechnology, biomaterials are constantly updated and applied in many areas. In environmental treatment, biotechnology is mainly divided into plant materials and microbial materials. Many algae and aquatic plants can be used for purification and repair. Among them, water hyacinth is quite effective in purification. It can turn harmful substances in the body into old leaves, and then, the leaves are removed by falling off, so as to replace the body. In the biological plant, the root system is used to absorb and fix the secretion, and then, it is purified. Second, the microorganism also has the adsorption function of many heavy metals. In the operation, sanitation gradually proliferates, and the selective removal efficiency of metals is very high. Coupled with the cultivation of biofilm, the increase of biofilm plays an important role in the adsorption mechanism. Zhao et al. pointed out that agricultural waste corn straw was burned at a high temperature to obtain corn straw biochar. Through the adsorption experiment of lead and cadmium in water, the heavy metal removal performance of high pyrolysis temperature biochar was investigated [9]. It treats waste with waste. Only two kinds of waste are used, which can produce a sharp tool for wastewater treatment. It has the advantages of a better energy-saving effect, multistage purification device, and so on. It can more effectively filter out harmful substances in the gas, which not only meets the requirements of environmental protection but also increases the income of investors.

### 4.2. The Role of Nanomaterials and Biofilm in Purifying Environmental Pollution

With the gradual enhancement of people's awareness of environmental protection, the problem of pollution has attracted much attention. Li et al. pointed out that with the gradual reduction of fresh water resources, the purification and treatment of sewage have become the most important thing at present. The water resources for urban watering and garden maintenance come from the secondary reuse of sewage treatment. Therefore, based on the multilevel biofilm as the starting point, the sewage technology of biofilm treatment, solve the current problem of sewage treatment [10]. Wang et al. proposed that the biofilm electrode reactor is a sewage treatment reactor, which combines the degradation function of the biofilm with the chemical reaction of the electrode, which can enhance the performance and will not be completely treated by the secondary pollution. The emergence of a three-dimensional biofilm electrode reactor, better than before, has increased the reaction system of spatial structure and improved the efficiency of the reactor [11]. Chen reported that as the sewage treatment speed and the use of freshwater resources break the balance, with the help of nanomaterials, the high catalytic efficiency and strong adsorption capacity greatly improve the speed of sewage treatment, which is widely used in water treatment engineering [12].

## 5. Comprehensive Analysis of Environmental Pollution and Treatment in the Development of Rural Cultural Industry

### 5.1. Effect Analysis of Different Materials on Environmental Pollution Control

With the development of industry and industrial construction, a large number of pollution have aggravated environmental pollution, which cannot be ignored for the destruction of the ecological environment and the impact of people's living environment; in this environment, the rise and development of nanomaterials provide a new purification treatment method for purifying the ecological environment and industrial development; the use of nanomaterials for the treatment of environmental pollution has the advantages of large specific surface area and more active sites, which is a better material for the treatment of pollutants; the following is an analysis of the treatment and purification effects of different materials on environmental pollution.

Table 1 shows that the effect of using general materials to purify the environment in rural industrial environmental purification is far less than that of nanomaterials and the role of nanomaterials in purifying environmental pollution is far greater than that of other common materials; Figure 2 is obtained by visual processing of the above data.

Figure 2 shows that nanomaterials mainly include natural nanomaterials and synthetic nanomaterials; in environmental treatment, the most widely used natural nanomaterials are clay minerals, such as kaolinite, which have good removal performance in heavy metals and fuel treatment; halloysite has a good application in pollutant removal and drug transportation; montmorillonite is also used as a nanosubstrate to combine with other nanomaterials to effectively remove the degradation of heavy metals and organic matter. Compared with natural nanomaterials, synthetic nanomaterials are purer in composition, diverse in structure, more prominent in performance, and more valuable in the treatment of environmental pollutants of different materials.

### 5.2. Comprehensive Effect Analysis under Different Environmental Pollution Control Technologies

In the application of modern technology, the use of biomaterials and biotechnology can effectively reduce or eliminate the generation of environmental pollution and pollutants caused by rural industrial production; the use of biomaterials, biofilm, and other technologies and materials has achieved good results in the treatment of wastewater pollution and wastewater microbial treatment methods; the obvious wastewater microbial treatment methods include the activated sludge method, biofilm method, anaerobic treatment method, microbial nitrogen removal process, and microbial phosphorus removal process; the following will analyze the comprehensive effect of environmental pollution control under different technologies.

Table 2 shows data on controlling environmental pollution and garbage caused by agricultural planting and animal husbandry, wastewater pollution, construction noise pollution, and research on several aspects of air pollution; under the application of biotechnology, the effect of purifying the environment is relatively high; visualize the data to get Figure 3.

Figure 3 shows that among the purification and treatment effects of several environmental pollutants, the environmental purification value under biotechnology is higher, which is more than one-third higher than that of the under traditional technology; it shows that the effect of purifying environmental pollution in biomaterials and biotechnology is better; biotechnology is not only effective in wastewater treatment but also will not produce secondary pollution in purifying waste gas and adsorbing and filtering air. In terms of solid waste treatment, it can also be transformed into agricultural organic fertilizers for secondary utilization, sustainable development, and utilization of resources, which greatly improves rural revitalization and industrial production.

### 5.3. Analysis of Coupling Degree of Different Materials for Purifying Environmental Pollution

Nowadays, based on the pursuit of a well-off level, national development emphasizes the harmonious development of urban and rural areas and common progress. As a part of the strategic development of rural revitalization, villages vigorously carry out creative industries in line with local characteristics on the basis of combining their own history, culture, and folk customs, which not only accelerates the rural modernization but also improves the intelligent life of residents and accelerates the development of rural economy; in addition, we should promote the comprehensive development of the country through local development. In the path of modern sustainable development, we should carry out rural green development roads and characteristic cultural industries and keep pace with the protection of the ecological environment and the purification of pollution.  Table 3 compares the coupling degree of environmental pollution purification with different materials:

Table 3 shows that the coupling degree of biomaterials in purifying environmental pollution is higher than that of traditional materials; the application and purification of biomaterials can better deal with and detect environmental pollution and avoid secondary pollution; data analysis showed that *t* < 10, *p* < 0.05; the data are statistically significant; visualize the data to get Figure 4.

Figure 4 shows that no matter the data before or after coupling, the treatment and purification of environmental pollution are relatively high when biomaterials are used; with the improvement of economic level, people pay more attention to the living environment. Environmental governance and purification are the primary tasks in the industrial development of rural development. The use of biotechnology can better avoid secondary pollution. Through the study of biomaterials and the intensity of biological purification of the environment, it provides value for the research and development of more efficient, lower energy consumption, and large-scale promotion of environmental governance technology.

## 6. Summary

In the development of modern urban and rural construction, firmly following the path of sustainable development and vigorously developing cultural and creative industries with rural characteristics is a necessary choice to promote the development of the rural economy with rural characteristics, and it is also an important measure to accelerate the modernization of agriculture and rural areas. It has driven the development and prosperity of the rural economy, but at the same time, in the purification of environmental pollution, we should actively use high-tech products and new environmental protection materials for industrial development, which is conducive to promoting the development of ecological balance and green economy. Biomaterials not only play an important role in environmental purification but also have gradually achieved great application results in modern industrial development and other fields, contributing more to the prosperity of the country. Through the role of biotechnology of biomaterials in environmental purification, it also better drives the economic benefits and environmental protection of rural areas, improves social benefits, and brings low-cost and high-yield effects to environmental governance. With the development and progress of biotechnology and materials, it will be conducive to the fundamental elimination of environmental pollution and destruction in the future. Turn the advantages of characteristic cultural resources into economic advantages, realize the organic unity of people's wealth and ecological beauty, and promote the formation of a green development mode and lifestyle, so as to realize the high-quality development of the rural economy.

## Figures and Tables

**Figure 1:** Environmental pollution trend in domestic rural cultural industry in 2014–2018.

**Figure 2:** Analysis of data on environmental pollution control by different materials.

**Figure 3:** Comprehensive analysis of environmental pollution control of rural cultural industry under different technologies.

**Figure 4:** Coupling degree of different materials to purify environmental pollution.

**Table 1:** Comparative analysis of environmental pollution control effects under different materials.

Group	Agricultural production pollution	Agricultural water pollution	Industrial air pollution	Construction noisepollution
General materials	42.23	46.29	50.11	48.21
Nanometer materials	63.02	65.36	68.25	64.27

**Table 2:** Comprehensive analysis of environmental pollution control of rural cultural industry under different technologies.

Group	Pollution control of planting andanimal husbandry	Water pollution control	Noise pollution control	Air pollutioncontrol
Traditional technology	35.26	41.11	38.26	42.69
Biotechnology	62.38	68.66	69.28	65.26

**Table 3:** Coupling degree of different materials to purified environmental pollution.

Group	Environmental pollution purification of rural cultural and creative industries (%)	
	Before coupling	After coupling
Traditional materials	32.69	43.65
Biological materials	52.69	69.92
*t*	8.235	8.653
*P*	0.026	0.023

## Data Availability

The data used to support the findings of this study are included within the article.
